RETRACTED

# Metaheuristic Optimization-Driven Novel Deep Learning Approach for Brain Tumor Segmentation

**DOI:** 10.1155/2022/2980691

**Published:** 2022-08-18

**Authors:** R. Kalpana, M. Anto Bennet, Abdul Wahab Rahmani

**Affiliations:** ^1^Department of Electronics and Communication Engineering, VelTech Rangarajan Dr. Sagunthala R&D Institute of Science and Technology, Avadi, Chennai, Tamil Nadu 600062, India; ^2^Isteqlal Institute of Higher Education, Kabul, Afghanistan

## Abstract

Brain tumor has the foremost distinguished etiology of high morality. Neoplasm, a categorization of brain tumors, is very operative in distinguishing and determining the tumor's exact location in the brain. Magnetic resonance imaging (MRI) is an efficient noninvasive technique for the anatomical examination of brain tumors. Growth tissues have a distinguishable look in MRI pictures in order that they are unit-wide used for brain tumor feature extraction. The existing research algorithms for brain tumors have some limitations such as different qualities, low sensitivity, and diagnosing the tumor at its stages. In this particular piece of research, an innovative method of optimization known as the procedure for lightning attachment algorithm (PLA) is used, and for the purpose of classification, a CNN model known as DenseNet-169 is applied. PLA was used in order to optimize the growth, and a network model known as the DenseNet-169 model was utilized in order to extract the various growth-optimization choices. First, the MR images of the brain were preprocessed to remove any outliers. Next, the Dense Net-169 CNN model was used to extract network choices from the MR images. In addition, it is used to execute the function of a classifier in order to identify the growth as either an aberrant growth or a traditional growth. In addition, the publicly benchmarked datasets that are widely utilized have validated the algorithmic rule that was granted. The planned system demonstrates the satisfactory accuracy in getting ready to on the dataset and outperforms many of the notable current techniques.

## 1. Introduction

Brain tumors are the foremost dreadful cancer among the various kinds of them. One of the most unpleasant types of cancer is a tumour, which has resulted in a massive population die-off [1]. Brain tumor needs precise analysis by the doctor that may categorize the tumor exactly [2]. Solely concerning, some kinds of brain tumors are cancerous, i.e., malignant. The tumor will impair the function of the brain either benign or malignant. It compresses the nerve and blood vessels and also causes many symptoms such as headaches perhaps severe, temperament changes, confusion, balance issues, nausea, difficulty in focusing, coordination, and concentration, numbness, weakness, and complication in sensory like hearing, vision, or speaking and seizures, and uncommon temporary state, amnesia, stumbling with thinking, speaking, and understanding languages [3].

RETRACTED

There are two sorts of tumours: benign and malignant. A tumour is occasionally treatable and is not considered malignant; however, a malignancy is harmful if it is not detected early. Tumors are among the various types of development that can be fatal and affect important brain components such as nerve tissue, white matter (WM), substantia grisea (GM), and liquid body material (CSF). This additionally damages the central nervous system [4]. Primary tumors will develop in the brain extent, and the tumors which develop apart from the brain extent are known as secondary tumors [3]. The tumor cells are also called neoplastic cells where they grow rapidly and divide in multiples more than the usual, or instead, they will not die [5]. One of the foremost common kinds of brain tumor is glioma. These gliomas emerge by the surrounding and nurture cells of glial cells, which also contain astrocytes, which are found in the brain, oligodendrocytes, and ependymoma cells [6]. The most common CNS tumor is low-grade glioma (LGG) and is categorized as grade-I and grade-II glial tumors, namely, oligodendodrogrioma and gangriomas pleomorphic xanthoastrocytoma. These were common mostly in pediatrics than adults. The least malignant and most common LGG is a pilocytic astrocytoma; by gross total research, overall survival can be >90-95% for about 5 years.  Figure 1(a) represents the epidemiology of LGG. Many patients have multiple progressions and recurrences depending on location and ability to resect. Then, the most aggressive and malignant glial tumor is high-grade glioma (HGG) which is classified as grade-III and grade-IV, and these were common mostly in adults than in pediatrics.  Figure 1(b) represents the epidemiology of HGG. HGG has a penurious survival outcome and is more resistant to therapy compared to LGG. The outcomes of HGG is universally poor showing 5-year overall survival is 15-20%. Nevertheless, recent analysis helps doctors move to victimization growth genetic science to higher classify gliomas. Individuals with a 5-year survival rate with a cancerous brain or system growth is three hundred and sixty-five days. The 10-year survival rate is concerning thirty-first. The 5-year survival rate for individuals younger than age fifteen is over seventy-fifth. For individuals aged fifteen to thirty-nine, the 5-year survival rate is over seventy-two. The 5-year survival rate for individuals aged forty and over is over twenty-first [7].

RETRACTED

The use of magnetic resonance imaging (MRI) in medical imaging allows for a good view of the body's soft tissues [5]. The positioning and size of these tumours in a brain magnetic resonance imaging (MRI) picture must be determined for diagnosis and therapy [8]. The most common types of MRI sequences are called T1-weighted and T2-weighted scans. When the TE and TR timings are kept relatively short, the resulting images are T1-weighted. The contrast and brightness of the image are mostly attributable to the characteristics of the T1 tissue. On the other hand, T2-weighted images are produced by employing TE and TR times that are significantly longer. The T2 properties of the tissue are primarily responsible for determining the contrast and brightness of these pictures. In this study, we present procedure for lightning attachment (PLA), a novel optimization approach inspired by lightning occurrences in which large quantities of electrical charges build up within the cloud. Lightning is created when the number of charges within a cloud increase, resulting in an increase in electrical intensity. Lightning can strike at any time, and it will erupt from a variety of locations [9].

This paper uses Dense Net Model as the basic structural unit feature extraction of the tumor and classifies the abnormal brain tumors in the LGG and HGG. When it comes to deep learning, CNNs (convolutional neural networks) are a type of deep neural network that is used to analyse graphical pictures. The dense convolutional network (Dense-Net), introduced in is a convolutional network where the layers are linked to all the further layers in the network. The Dense-Net is used for accurate feature extraction of the image. In our proposed model, Dense net 169 is used as a feature extractor. The Dense-Net architecture has been proposed in recent years, and work on standard datasets has shown it to be substantially deeper, more accurate, and efficient than most architectures. Its dense interconnections between layers are proposed to encourage feature reuse [10].

### 1.1. Contribution of the Paper

- We use BraTS 2016, 2017, and BraTS 2018 datasets to be used in the training and validation phases
- The brain tumor features were extracted and classified by utilizing DenseNet-169 for obtaining deeper and more generic features
- We propose a novel method named lightning attachment procedure algorithm for feature selection
- The performance measures are evaluated with optimization performance

The remainder of the paper is structured as follows: Section 2 is dedicated to related work. The preprocessing method and the phase of scheme are explained in Section 3. The experimental results of the advanced model is explain in Sections 4 and 5. Finally, in Sections 6, the findings and future work are discussed.

RETRACTED

## 2. Related Works

Brain tumor optimization is embraced for tumor detection due to high mortality, and many researchers are floundering to diagnose brain tumors at early stages using several machine learning architectures. The very first step for brain tumor optimization is preprocessing Kumar (2020) [5] developed a deep learning algorithm that has been tuned called Dolphin-SCA correlated with D-CNN for effective classification and segmentation of brain tumor. After preprocessing, the segmentation is passed out by a vague deformable blending model with dolphin-SCA. And on power LDP and statistical characteristics, the feature extraction method is carried out. These features are used in D-CNN for the sorting of brain tumor with D-SCA and were compared with the BraTS and Sim BraTS datasets. However, for effective treatments, the accuracy of the current model should be improved. Brain tumour segmentation approaches based on classical image processing and machine learning are not optimal enough among the currently suggested brain segmentation methods. After preprocessing feature extraction is the vital procedure which is done by Yin et al. (2020) [8], a novel metaheuristic-based technique for brain tumour early detection background removal, feature extraction, and classification using a multilayer perceptron neural network are the three key aspects of the proposed technique. The best selection of features and classification stages is achieved using an updated model of the whale optimization method based on chaos theory and logistic mapping approach. Furthermore, Alagarsamy et al. (2021) [11] used a spatially constrained fish school optimization method (SCFSO) and an interval type-II vague logic system to address brain tumour abnormalities. SCFSO and IT2FLS can intervene and investigate large datasets and complicated cancers. The suggested approach provides a distinct separation of the tumour and nontumor regions, allowing for treatment preplanning. Huge database requirements and high computational time still pose a problem for deep learning. So, a lot of work is done for feature extraction in order to forecast the occurrence of a brain tumour. Deb and Roy (2021) [12] recommended a system to identify picture normalcy and abnormality; we used an adaptive fuzzy deep neural network with frog leap optimization. Classification is done by AFNN, and segmentation is done using adaptive flying squirrel algorithms. The accuracy gained by the proposed system is 99.6%. Additionally, various authors have proposed different feature extraction models to classify brain tumors. For the identification of brain tumours, Sharif et al. (2019) [13] designed a swarm optimization with a blending of characteristics which was used. In the initial stage, the head is taken out by the BSE technique. Then, the image is fed to PSO for segmentation. For feature selection, a genetic algorithm is used to extract LBP and deep features from segmented pictures. At last, the classification of tumor kinds is done using ANN and is compared with the RIDER and BraTS datasets.

RETRACTED

Because of the time necessary for the training process, this suggested system has certain disadvantages, including a long processing time and decreased accuracy. Later, Cristin et al. (2021) [14] created an excellent tumour classification algorithm called fractional-chicken swarm optimization (fractional-CSO). To improve the accuracy, chicken swarm is combined with a derivative factor. The MR pictures have been preprocessed, and the features have been retrieved efficiently. The tumour classification security level is achieved utilising deep recurrent neural networks that are trained using the suggested fractional CSO technique and have an accuracy of roughly 93.35 percent. The conventional methods lack accuracy in segmentation due to the complex spatial variation of tumors. Furthermore, Shivhare and Kumar (2021) [4] proposed the MLP (multilayer perceptron) to improve the accuracy of segmentation of brain tumours, to improve the accuracy of segmentation of brain tumours, and to improve the accuracy of segmentation of brain tumours. For this, three metaheuristic optimization algorithms GWO, AEFO, and SMO have been used. Grounded on the voting, a majority three models have been combined. The three brain tumor regions are segmented by different magnetic resonance modalities. The proposed system uses the BraTS dataset and can achieve 92% of DSC. Rammurthy and Mahesh (2020) [2] experimented with an automatic tumor classification model. This paper an optimized Whale Harris Hawks Optimization technique is used. The dissection process is done using cellular automata and rough set theory. Some features like size, LOOP, mean, variance, and kurtosis are extracted from segments. Detection done using D-CNN, wherein the training is done using the proposed model, is designed by WOH and HHO Algorithm. Different strategies for brain tumour classification have been created in the literature and, however, owed to inaccuracy, then inadequate result making the prevailing techniques have failed to give enhanced classification. Besides, Vilas et al. (2020) [10] proposed spontaneous brain tumor dissection using Dense Net. In this project, we recommend a Dense Net architecture for automatic segmentation based on CNN. The performance of Dense Net architecture against that of U-net is utilized, and the drawn analysis is compared with the BraTS dataset.

RETRACTED

## 3. Methodology Proposed

Skull scripting is adopted as a preprocessing in our proposed model, followed by Dense Net-169 for feature extraction and classification. Procedure for lightning attachment has been used to execute a feature selection step prior to categorization (PLA). The above procedures are used in the BraTS datasets from 2016, 2017, and 2018. The architecture for the suggested model is shown in Figure 2.

### 3.1. Dataset Description

For the purpose of training and validation of the architecture that has been proposed, three datasets were used in this study. BraTS 2016, BraTS 2017, and BraTS 2018, respectively, were chosen as the datasets. Each database contains ground-truth photos for four distinct classes, including Flair, T1CE, T1, and T2. The datasets are divided into two distinct modes: LGG and HGG, with each distinct mode containing four stage tumours (T1-weighted, T1CE, T2-weighted, and flair) [15]. To resolve disparities, the data is removed from the skull, aligned to suit an anatomical template, and resampled at 1 mm^3^ resolution. A volume (dimension) of 240∗240∗155 is assigned to each sequence [16]. All photos have anisotropic resolutions that are resampled to become isotropic. The 60% flair and T1CE photos, as well by using this picture, ground truth images are utilised to train a CNN model for the disunion technique. The remaining 40% of photos, from both classes, and 100% of T1 and T2 are used in the testing phase [1]. The BraTS datasets' training validation is shown in Table 1.  Figure 3 shows a selection of photos from the BraTS collection.

### 3.2. Skull Stripping as Preprocessing

Skull striping is the process of removing nonbrain structures and undesired picture sections from a scanned image in order to obtain the image necessary for tumour identification. The brain, scalp, skull, and dura are all visible in the photograph. With the use of a cerebrospinal fluid rim, you can separate the undesired components (CSF). Intensity thresholding and morphological operations can be used to remove the skull and acquire the requisite brain region for tumour identification. Allow the input picture to be epitomised as a collection of pixels with intensity values at relevant locations in the image.

(1) $$\begin{array}{c} \text{Let }Ip=Ip1,Ip2,Ipn=Ipn=Ipn=Ipn=Ipn=Ipn=Ipn=Ipn. \end{array}$$

In the case of IP1, the intensity levels of pixels 1 to *n* are represented by the integer *Ipn*. And *np* stands for the total number of pixels in a picture. Let us say the intensity threshold is *T*, and the circumstance for removing pixels extracted from the picture is that the intensity of those pixels is less than *T*. Pixels that match this requirement are normally used to denote thin connections. The technique meets two conditions. The first is that nonbrain structures should be only weakly connected to the brain. The mask formed by intensity thresholding should also preserve as much brain as possible undamaged. Setting the proper threshold number is critical in this case, since setting it too low might result in the inclusion of garbage, which is undesired. Threshold levels that are too high can assist distinguish between brain and nonbrain structures, but they come at the expense of brain function.

RETRACTED

We now have the requisite brain picture, which must be improved to make it suitable for the tumour identification procedure. We employ morphological procedures to do this. It also aids in the elimination of tight connections [18].

### 3.3. Feature Extraction

By directly integrating all layers with the same feature sizes, DenseNet is able to solve the problem of gradient vanishing, which occurs frequently in deep CNN. The multilayer architecture of the DenseNet-169 is seen in Figure 3. The most compelling justification for utilising DenseNet as a feature extractor is due to the fact that as you delve further into the network, you will become aware of an increasing number of general features. The method for the extraction of features was carried out with the assistance of a densely connected convolutional neural network (DenseNet-169) that had been trained in advance. The variant that was used in this work was trained with the use of the ImageNet dataset, which is a large dataset that is accessible to the public.

In order to create the DenseNet169 architecture, one layer of complexity and amalgamation is placed at the beginning, followed by three conversion layers and four dense blocks. The classification layer comes after these previous stages have been completed. The first convolutional layer performs 7∗7 intricacies when stride 2 is used, and this is followed by a maximum pooling of 3∗3 when stride 2 is used. After then, there is a dense block in the network that is surveyed by three sets. Within each set is a conversion layer, and then, there is a dense block. Conversion layers are the names given to the layers that can be found between thick blocks. A batch normalisation layer and a 1∗1 convolutional layer come first in each of the network's conversion layers. Next comes a 2∗2 average pooling layer with a stride of 2 and finally comes a stride of 2.

As previously stated, there are four dense blocks, each of which has two intricacy layers, the first of which is of 1∗1, and the second of which is of size 3∗3. The four dense blocks of the DenseNet169 design pretrained on ImageNet are 6, 12, 32, and 32 pixels in size. Following this is the sorting layer, which does overall average pooling of 77% and finally followed by fully connected layer that uses “softmax” as the activation [19].

RETRACTED

### 3.4. Classifier

In recent years, CNN has made significant improvement in a number of areas, including picture categorization. This is due to the fact that CNN networks are one of the most accurate technologies currently available for detecting characteristics in input pictures.

Intricacial layers, initiation layers, set normalisation layer, and amalgamating layers are used for feature extraction in Dense Net-169, while dropout layers are utilised for classification.

- Compressed layers, also known as completely linked layers, comprise numerous neurons or units, with the last thick layer has the same number of neurons as the number of categories. The activation layer is placed after each dense layer. The activation function used to the output of the final dense layer differs significantly from the sigmoid or softmax function used in the previous dense layers. In multiclass classification tasks, each category is assigned decimal probabilities using the Softmax function, with the target category having the greatest probability. The following formula is used to calculate the softmax of *i*th output unit

(2) $$\begin{array}{c} {\hat{y}}_{i}=\frac{e^{x_{i}}}{\sum_{i}^{N}e^{x_{i}}},\text{ For }i=1,2,3,\cdots ,N, \end{array}$$

where *x*_*i*_ is the output of the *i*th dimension, *N* is the no. of dimensions, and ${\hat{y}}_{i}$ is the probability associates with the *i*th category.

During forecasting, a sample is assigned to the category with the highest likelihood, as indicated below.

(3) $$\begin{array}{c} {\hat{y}}_{i}=\underset{i\in \left[1,N\right]}{\max}{\hat{y}}_{i}. \end{array}$$

In binary classification problems, the sigmoid function is employed. It accepts any real number between 0 and 1 and returns a result that falls inside that range. The following equation is used to compute it numerically:

(4) $$\begin{array}{c} \text{Sigmoid}\left(X\right)=\frac{1}{1+e^{-x}}. \end{array}$$

(ii) Dropout layers are a regularisation method used only during network training to prevent overfitting by temporarily removing a subsection of the inputted neurons and their connections from the thick layer before them. Except the last layer, which yields category-specific probabilities, the dense layers are normally surveyed by a loafer layer

RETRACTED

### 3.5. Feature Selection: Procedure for Lightning Attachment (PLA)

The suggested algorithm and its source of inspiration are shown in this section. Lightning is caused by an increase the total number of charges stored in the cloud, which results in a surge in electrical intensity. Precipitous will airstrike, and it may hit several times.

The four phases of attachment to precipitous technique are as follows: (1) breakup of air at the cloud's surface, (2) descendant motion of the lightning channel, (3) ascendant leader expansion, and (4) ultimate hit location [9].

#### 3.5.1. Creativity

The four processes of lightning attachment are as follows: (1) air disintegration on the cloud surface, (2) descending exodus of the precipitous channel, (3) the formation and spread of rising leaders from the ground earthed objects, and (4) final leap. These steps are detailed in this article.

*(1) Cloud Edge Air Breakdown*. As seen in Figure 4, the cloud's charge may be broken down into three pieces: a large amount of negative charge in the cloud's lower half, a large amount of affirmative charge in the cloud's superior part, and tiny amount of affirmative charge in cloud's bottom portion. The potential between the charge centres grows as the number of these charges grows, and it is possible for the negative charges to separate from the large positive charge section or the little positive charge component. As a result of this breakdown, power gradient near the cloud's edge rises, lightning forms, and a massive amount of electrical energy (mainly negative charge) flows toward the earth. Lightning may originate from several points, as evidenced by high-speed images of genuine lightning strikes [20].

*(2) Effort of the Downhill Leader Headed for the Earth*. The precipitous approaches the ground in an ongoing motion as the air breakdown occurs near the cloud's edge. The precipitous comes to a halt after each stride, then continues in one or more different directions towards the earth. To comprehend this technique, envision a hemisphere underneath the leader tip with the midpoint of the leader tip and the ambit of the next step length after each step. On the surface of this hemisphere, there are several potential jump places to choose from. The next jump point is chosen at random, however, a place, with a greater electrical field value; it is more likely that the line connecting the leader tip and the matching point will be picked.

*(3) Fading Branches*. The charge of the upper most division is allocated into innovative divisions if there are more than one point for the following lightning jump. The same technique is followed for all new branches, resulting in the formation of new branches. When the charge on a branch falls below critical value (IC), there is no decomposition of air and so no additional movement. As a result, this branch would vanish.

*(4) Propagation of Upward Leaders*. Clouds indicate that there is a massive negative charge above the ground. Positive charges clump together on the earth surface or on an earthed item underneath the cloud as a result of this. The intense electric field produces air breakup in the sharp points; thus, the upward leader begins there and spreads across the air. These upper leads accelerate their approach to the descending leader as it reaches the earth. The ascending leaders likewise go through the branching and branch fading process.

*(5) Final Leap (3.5.1.5). (Striking Point Determination)*. The ultimate jump happens whenever an ascending leader reaches a descending leader, and the striking point is the place where the upward leader began. All other branches vanish in this condition, and the cloud's charge is absorbed through this route [21].

*(6) The PLA Algorithm*.

RETRACTED

**Step 1 .**

Trial spots.

The trial locations indicate the downward leaders' beginning points, which is obtained as follows:

(5) $$\begin{array}{c} X_{ts}^{i}=X_{\min}^{i}+\left(X_{\max}^{i}-X_{\min}^{i}\right)*\mathrm{rand}. \end{array}$$

The initial trial locations are denoted by *X*_*ts*_^*i*^. The control variable's lowest value is *X*_min_^*i*^, and its maximum value is *X*_min_^*i*^. rand is a random number between 0 and 1. For the first places, the fitness function is determined as follows:

(6) $$\begin{array}{c} F_{ts}^{i}=\text{obj }\left(X_{ts}^{i}\right). \end{array}$$

**Step 2 .**

Determination of the next leap.

The fitness values are calculated by averaging all of the original points:

(7) $$\begin{array}{c} X_{\text{avr}}=\text{mean}\left(X_{\text{ts}}\right),\\ F_{\text{avr}}=\text{obj}\left(X_{\text{avr}}\right). \end{array}$$

The average point is denoted by *X*_avr_, and the neutral purpose of the average point is denoted by *F*_avr_. As previously stated, the lightning has multiple paths where it jumps to the next highest optional point. A random solution *j* (potential point) is chosen to update the point I so *i* ≠ *j*. The acquired answer is then compared to the possible solution. As a result, the following formula may be used to determine the next jump:

(8) $$\begin{array}{c} X_{\text{ts}\_\text{new}}^{i}=X_{\text{ts}}^{i}+\mathrm{rand}*\left(X_{\text{avr}}+X_{\text{PS}}^{j}\right)\text{IF}{\text{F}}_{j}<F_{\text{avr}},\\ X_{\text{ts}\_\text{new}}^{i}=X_{\text{ts}}^{i}-\mathrm{rand}*\left(X_{\text{avr}}+X_{\text{PS}}^{j}\right)\text{IF}{\text{F}}_{j}>F_{\text{avr}}. \end{array}$$

**Step 3 .**

RETRACTED

Fading of sections.

If the critical value is smaller than the electric field of the new test point, the branch will stay continuous; otherwise, it will fade, as shown in the following diagram.

(9) $$\begin{array}{c} X_{\text{ts}}^{i}=X_{\text{ts}\_\text{new}}^{i}\text{IF}{\text{F}}_{\text{ts}\_\text{new}}^{i}<F_{\text{ts}}^{i}. \end{array}$$

In this procedure, test points are run, and the first stage's leftover points are moved down.

**Step 4 .**

Rising march of the leader.

The ascending leader, which is spread throughout the canal significantly, moves the points up in this operation. As a result, an exponent operator looks like this:

(10) $$\begin{array}{c} S=1-\left(\frac{t}{t_{\max}}\right)*\exp\left(-\frac{t}{t_{\max}}\right). \end{array}$$

If *t* is the number of iterations, and *t*_max_ is the maximum number of iterations, and next leap is determined by the channel's charge, the next point is as follows:

(11) $$\begin{array}{c} X_{\text{ts}\_\text{new}}^{i}=X_{\text{ts}\_\text{new}}^{i}+\mathrm{rand}*s*\left(X_{\text{best}}^{i}-X_{\text{worst}}^{i}\right), \end{array}$$

where *X*_best_^*i*^ and *X*_worst_^*i*^ are the best and the worst solutions among the populations.

**Step 5 .**

No returns of lightning.

When the down and up leaders get together, and the striking spot is assigned, the lightning operation comes to a halt [9].

## 4. Performance Assessments

To assess the recommended ML model with optimization performance, performance metrics including accuracy, error rate, sensitivity, specificity, and *F*1-measure are employed.

True positives (TP) are instances in which the ground truth image's tumour (1) data point is accurately identified as the segmented image's tumour (1) data point.

True negatives (TN) occur when a ground truth image's nontumour (0) data point is accurately tagged as a segmented image's nontumour (0) data point.

False positives (FP) happen when a ground truth image's nontumour (0) data point is incorrectly identified as a segmented image's tumour (1) data point.

False negatives (FN) are when the ground truth image's tumour (1) data point is accurately tagged as the segmented image's nontumour (0) data point.

The number of positive and negative data points divided by the total number of data points is known as accuracy

(12) $$\begin{array}{c} \text{ Accuracy}=\frac{\left(\text{TP}+\text{TN}\right)}{\left(\text{TP}+\text{TN}+\text{FP}+\text{FN}\right)}*100. \end{array}$$

The ratio of genuine positives to positive calls is known as precision or specificity. Positive predictive rate (PPR):

(13) $$\begin{array}{c} \text{Specificity}=\frac{\text{TP}}{\text{TP}+\text{FP}}. \end{array}$$

The chance of a positive test if the patient has a tumour is known as recall or sensitivity. It is also known as the true-positive rate:

(14) $$\begin{array}{c} \text{Sensitivity}=\frac{\text{TP}}{\text{TP}+\text{FN}}. \end{array}$$

RETRACTED

## 5. Result and Discussion

### 5.1. Contrast

The proposed PLA-Deep CNN mechanism is associated to four current techniques: (i) Dolphin Echolocation-based Sine Cosine Algorithm +fuzzy-based Naive Bayes (Dolphin-SCA+FNB) [5], (ii) DWT-deep belief network (DBN) (DWT+DBN) [22], (iii) Bayesian HCS-multi-SVNN [23], and (iv) Fractional—the comparison study for BraTS 2016, 2017, and 2018 data is shown in Tables 2–4.

#### 5.1.1. Using the BraTS 2016 Information, a Comparative Study Was Conducted

- Variation of data analysis for training

Using the BraTS 2016 database with different training data percentages, the recommended PLA-Deep CNN is compared to current approaches like Dolphin-SCA + FNB, DWT + DBN, Bayesian HCS-multi-SVNN, and Fractional CSO + DRNN in relations of specificity, compassion, and precision. The specificity analysis findings for various training data percentages are shown in Figure 5(a). Dolphin-SCA + FNB, DWT +DBN, Bayesian HCS-multi-SVNN, and Fractional CSO +DRNN all have specificity scores of 93.57 percent, 94 percent, 93.89 percent, and 94 percent, respectively, with 90 percent training data. The proposed PLA-based Deep CNN technique has a high specificity, which means it can recognise negatives more accurately. The findings of the sensitivity parameter analysis utilising the BraTS 2016 database are shown in Figure 5(b). When the training data percentage is 70, the relevant sensitivity values measured by Dolphin-SCA + FNB, DWT +DBN, Bayesian HCS-multi-SVNN, Fractional CSO +DRNN, and suggested PLA-based Deep CNN are 95.94 percent, 93 percent, 92.59 percent, 93 percent, and 95.9 percent.  Figure 5 depicts the precision parameter analysis by the BraTS 2018 record (c). The precision values assessed by Dolphin-SCA + FNB, DWT +DBN, Bayesian HCS-multi-SVNN, Fractional CSO +DRNN, and the suggested PLA-based Deep CNN are 93.35 percent, 91.38 percent, 90.98 percent, 93.75 percent, and 94 percent, respectively, once the exercise data proportion is 50. Among the existing techniques, the recommended PLA-based Deep CNN has the maximum accuracy, showing that it is capable of reliably recognising the tumorous region.

(ii) Variation of *K*-Fold analysis

Figure 5 depicts a qualified analysis plot based on specificity, understanding, and precision metrics by the BraTS 2016 record for different *K*-Fold values.  Figure 6 depicts the results of a specificity examination for *K*-Fold values vacillating from 2 to 6. (a). For *K* − Fold = 2, the specificity standards measured by Dolphin-SCA + FNB, DWT +DBN, Bayesian HCS-multi-SVNN, and Fractional CSO +DRNN are 0.767, 0.765, 0.691, 0.702, and 0.863, respectively.  Figure 6 depicts the results of the sensitivity parameter analysis using the BraTS database (b). Dolphin-SCA + FNB, DWT +DBN, Bayesian HCS-multi-SVNN Fine Tuned CNN Fractional CSO +DRNN, and suggested PLA-based Deep CNN exhibit sensitivity values of 0.895, 0.958, 0.927, 0.965, and 0.981 when *K* − Fold = 2.  Figure 6 depicts the precision parameter analysis using the BraTS record. (c). When *K*-Fold is equal to 4, the precision values assessed by Dolphin-SCA + FNB, DWT +DBN, Bayesian HCS-multi-SVNN Fine Tuned CNN Fractional CSO +DRNN, and suggested PLA-based Deep CNN are 0.796, 0.824, 0.795, 0.875, and 0.907.

(iii) ROC analysis

Once FPR is 0.3, the analogous TPR standards restrained by Dolphin-SCA + FNB, DWT +DBN, Bayesian HCS-multi-SVNN, Fractional CSO +DRNN, and projected and proposed PLA-based Deep CNN are 0.905, 0.742, 0.712, 0.84, and 0.943, respectively. Furthermore, the suggested PLA-based Deep CNN outperforms the FPR = 0.8, 0.9, 1 for identifying tumour and nontumour areas with a TPR of 1.

RETRACTED

#### 5.1.2. Using the BraTS 2017 Information, a Comparative Study Was Conducted

- Variation of data analysis for training

The recommended PLA-based Deep CNN is compared to current approaches such as Dolphin-SCA + FNB, DWT +DBN, Bayesian HCS-multi-SVNN, and Fractional CSO +DRNN in terms of specificity, compassion, and precision using the different training data percentages from the BraTS 2017 database.  Figure 7 depicts the findings of a research on specificity for different training data percentages (a). Dolphin-SCA + FNB, DWT +DBN, Bayesian HCS-multi-SVNN, and Fractional CSO +DRNN have specificity values of 94.9 percent, 95 percent, 94.68 percent, and 95 percent, respectively, whereas suggested PLA-based Deep has a specificity of 95.7 percent with 90% training data. The suggested PLA-based Deep CNN approach has a high specificity, and as a result, it has a better capacity to properly recognise negatives. The sensitivity parameter analysis utilising the BraTS 2017 database is shown in Figure 7(b). The sensitivity values determined by Dolphin-SCA + FNB, DWT +DBN, Bayesian HCS-multi-SVNN, Fractional CSO +DRNN, and suggested PLA-based Deep CNN are 96.8%, 94.5 percent, 94.5 percent, and 96.2 percent, respectively, once the physical activity data percentage is 70%. The accuracy parameter analysis utilising the BraTS 2018 database is shown in Figure 7(c). The precision values assessed by Dolphin-SCA + FNB, DWT +DBN, Bayesian HCS-multi-SVNN, Fractional CSO +DRNN, and suggested PLA-based Deep CNN are 94.5 percent, 92.88 percent, 91.90 percent, 92.67 percent, and 95 percent, respectively, when the training data percentage is 50. The suggested PLA-based Deep CNN has all the known techniques and has the highest accuracy, indicating that it is capable of accurately identifying the tumorous portion.

(ii) Variation of *K*-Fold analysis

For varied *K*-Fold values, employing the BraTS 2018 database, Figure 8 depicts a relative analysis plot using specificity, sensitivity, and accuracy measures.  Figure 7 shows the results of a specificity study for *K*-Fold values ranging from 2 to 6 (a). Dolphin-SCA + FNB, DWT +DBN, Bayesian HCS-multi-SVNN, and Fractional CSO +DRNN have specificity values of 0.798, 0.772, 0.708, 0.691, and 0.871, respectively, while the suggested PLA-based Deep CNN has a specificity of 0.842 for *K* − Fold = 2. The results of the sensitivity parameter analysis utilising the BraTS database are shown in Figure 8(b). When *K* − Fold = 2, the sensitivity values of Dolphin-SCA + FNB, DWT +DBN, Bayesian HCS-multi-SVNN, Fractional CSO +DRNN, and suggested PLA-based Deep CNN are 0.901, 0.962, 0.938, 0.942, and 0.971, respectively. Figure 8 shows the results of the accuracy parameter study using the BraTS database (c). When *K* − Fold = 4, the accuracy scores of Dolphin-SCA + FNB, DWT +DBN, Bayesian HCS-multi-SVNN, Fractional CSO +DRNN, and the suggested PLA-based Deep CNN are 0.881, 0.831, 0.801, 0.891, and 0.913, respectively.

(iii) ROC-based analysis

TPR values measured by Dolphin-SCA + FNB, DWT +DBN, Bayesian HCS-multi-SVNN, Fractional CSO +DRNN, and proposed PLA-based Deep CNN are 0.912, 0.735, 0.831, 0.85, and 0.951, respectively, when FPR is 0.3. Furthermore, the suggested PLA-based Deep CNN outperforms the FPR = 0.8, 0.9, and 1 in categorising tumour and nonneoplastic areas with a TPR of 1.

RETRACTED

#### 5.1.3. Using the BraTS 2018 Information, a Comparative Study Was Conducted

- Variation of the training data analysis

In Figure 9, the suggested PLA-based Deep CNN is compared to current approaches such as Dolphin-SCA + FNB, DWT +DBN, Bayesian HCS-multi-SVNN, and Fractional CSO+DRNN in terms of specificity, compassion, and precision using the BraTS 2018 database for different training data percentages. Figure 9 shows the specificity analysis for different training data percentages (a). Dolphin-SCA + FNB, DWT +DBN, Bayesian HCS-multi-SVNN, and Fractional CSO +DRNN had specificity values of 95.3 percent, 96 percent, 95.09 percent, and 96 percent, respectively, and recommended PLA-based Deep 97 percent for 90 percent training data. The suggested PLA-based Deep CNN approach has a high specificity, which means it has a better capacity to properly recognise negatives.

Using the BraTS 2018 database, the analysis in terms of the sensitivity parameter is shown in Figure 9(b). When the training data percentage is 70%, the sensitivity values assessed by Dolphin-SCA + FNB, DWT +DBN, Bayesian HCS-multi-SVNN, Fractional CSO +DRNN, and proposed PLA-based Deep CNN are 97.7%, 95.29 percent, 95 percent, and 98 percent, respectively. Using the BraTS 2018 database, the accuracy parameter analysis is shown in Figure 9(c). The equivalent accuracy values measured by Dolphin-SCA + FNB, DWT +DBN, Bayesian HCS-multi-SVNN and Fractional CSO +DRNN and suggested PLA-based Deep CNN are 95.3 percent, 93.20 percent, 92.56 percent, 93.35 percent, and 96.8 percent when the training data percentage is 50. Among the available approaches, the suggested PLA-based Deep CNN has the best accuracy, indicating that it is capable of accurately identifying the tumorous portion.

(ii) Variable *K*-Fold analysis

Using the BraTS 2018 database, Figure 10 shows a relative investigation plan created on specificity, compassion, and precision characteristics for varied *K*-Fold values. Figure 10 shows the results of a specificity study for a range of *K*-Fold values from 2 to 6. (a). Dolphin-SCA + FNB, DWT +DBN, Bayesian HCS-multi-SVNN, and Fractional CSO +DRNN have specificity values of 0.801, 0.795, 0.724, and 0.882, respectively, whereas the suggested PLA-based Deep CNN has a specificity of 0.851 for *K* − Fold = 2. Using the BraTS database, the examination in relations of the understanding parameter is shown in Figure 10(b). Dolphin-SCA + FNB, DWT +DBN, Bayesian HCS-multi-SVNN, Fractional CSO +DRNN, and projected PLA-based Deep CNN have sensitivity values of 0.923, 0.971, 0.942, 0.959, and 0.981 when *K* − Fold = 2. Figure 10 shows the results of the precision parameter study using the BraTS record (c). When *K*-Fold is equal to 4, the precision values assessed by Dolphin-SCA + FNB, DWT +DBN, Bayesian HCS-multi-SVNN Fine Tuned CNN Fractional CSO +DRNN, and proposed PLA-based Deep CNN are 0.892, 0.843, 0.825, 0.893, and 0.924, respectively.

(iii) ROC-based analysis

After FPR is 0.3, the comparable TPR morals assessed by Dolphin-SCA + FNB, DWT +DBN, Bayesian HCS-multi-SVNN, Fractional CSO +DRNN, and suggested PLA-based Deep CNN are 0.9276, 0.742, 0.845, 0.86, and 0.964. Furthermore, the suggested PLA-based Deep CNN outperforms the FPR = 0.8, 0.9, and 1 in categorising tumour and nonneoplastic areas with a TPR of 1.

In this paper, a novel enhanced PLA is suggested as a complete technique for brain tumour classification based on optimum feature selection. For the validation of the proposed technique, two BraTS datasets were employed. The preprocessing technology is intended to aid in the categorization of brain tumours in brain imaging. Cristian et al. (2021) presented fractional-chicken swarm optimization (fractional-CSO) as a useful categorization approach. The cancer categorization is carried out once the brain pictures have been preprocessed and the characteristics retrieved efficiently. Using a simulated BraTS dataset, we achieved accuracy, specificity, and sensitivity of 93.35, 96, and 95 percent. For brain tumour diagnosis utilising MR images, Rammurthy and Mahesh (2020) introduces Whale Harris Hawks Optimization (WHHO), an optimization-driven approach. Maximum accuracy, sensitivity, and specificity for the proposed WHHO-based Deep CNN were 0.816, 0.974, and 0.791, respectively. On a set of benchmark cases, PLA's experimental findings are compared to those of other common optimizers, and the results are confirmed. According to the comparative results in the tables, employing the suggested technique for improving picture feature selection and ML classification produces good results when compared to existing optimization methods.

RETRACTED

## 6. Conclusion

In this study, the procedure for lightning attachment (PLA) plus support vector machine (SVM) classifier is proposed as a brain tumour classification method for finding cancer locations from MRI data. Both of these classification methods are combined into one. Both the training and the validation of our proposed architecture made use of the datasets that we acquired, which were referred to as BraTS 2017 and BraTS 2018. Skull stripping, also known as the elimination of nonbrain structure and undesirable aspects of an image obtained from a scanned photograph in order to obtain the necessary imaging for the identification of a tumour, is a technique that is used to remove components that are not requested. In this particular scenario, the preprocessor known as “skull stripping” is utilised. The characteristics are extracted by DenseNet-169, which then produces features that are more general for the deeper network. Following that, the procedure for lightning attachment is used to the feature selection process. This population-based strategy got its start because of the physical phenomena that occur during the lightning attachment technique. These phenomena include air interruption, descending leader movement, ascending leader inception and dispersion, and ultimate leap. Our research utilised a classifier known as a sustainment vector machine (SVM), which brings us to the next stage of the process, which is classification. Because it is a binary classifier that is based on supervised learning, it differentiates between two classes by building a hyperplane in high-dimensional feature space. This allows it to process information in a more efficient manner. The reliability of the system may be improved by increasing the amount of data points. The process of accurately classifying things may lead to the discovery of other features that are significant in this regard. This computerised method could also be used to categorise other brain diseases in addition to other medical photographs of various pathological situations, types, and states of disease.

RETRACTED

## Figures and Tables

**Figure 1:** Epidemiology of LGG and HGG.

**Figure 2:** Architecture for suggested model.

**Figure 3:** A selection of pictures from the Multimodal Brain Dataset (BraTS) [17].

**Figure 4:** The formation of charges in the cloud [9].

**Figure 5:** Analysis of specificity, sensitivity, and accuracy using the BraTS 2016 database. (a) Specificity, (b) sensitivity, and (c) accuracy.

**Figure 6:** Using the BraTS 2016 database, analysis by altering *K*-Fold. (a) Specificity, (b) sensitivity, and (c) accuracy.

**Figure 7:** Analysis utilising the BraTS 2017 database with different training data. (a) Specificity, (b) sensitivity, and (c) accuracy.

**Figure 8:** Analysis utilising the BraTS 2017 database and adjusting *K*-Fold. (a) Specificity, (b) sensitivity, and (c) accuracy.

**Figure 9:** Training data analysis utilising the BraTS 2018 database. (a) Specificity, (b) sensitivity, and (c) accuracy.

**Figure 10:** Using the BraTS 2018 database, examine the effects of changing *K*-Fold. (a) Sensitivity, (b) accuracy, and (c) specificity.

**Table 1:** Training and validation datasets for the BraTS system.

Dataset	Description
BraTS-2016 [13]	Each has 220 aberrant higher-grade glioma (HGG) photos and 54 normal lower-grade glioma (LGG) images.
BraTS 2017 [1]	There have been a total of 431 examples in total, 285 training cases (210 HGG and 75 LGG) and 146 testing cases (both HGG and LGG) were included in the study.
BraTS 2018 [1]	There has been a total of 476 examples in total, 285 training cases (210 HGG and 75 LGG) and 191 testing cases for both HGG and LGG were included in the study.

**Table 2:** Discussion of the BraTS 2016 dataset in comparison.

Techniques	Acc (%)	Spec (%)	Sens (%)
Dolphin SCA+ FNB	93.35	93.57	95.94
DWT+DBN	91.38	94	93
Bayesian HSC multi-SVNN	90.98	93.89	92.59
Fine-tuned CNN	90.63	93.25	92.89
Fractional CSO	93.75	94	93
PLA + Dense Net-169	94	95.2	95.9

**Table 3:** Discussion of the BraTS 2017 dataset in comparison.

Techniques	Acc (%)	Spec (%)	Sens (%)
Dolphin SCA+ FNB	94.5	94.9	96.8
DWT+DBN	92.88	95	94
Bayesian HSC multi-SVNN	91.90	94.68	93.95
Fine-tuned CNN	91.56	94.42	93.58
Fractional CSO	92.67	95	94
PLA + Dense Net-169	95	95.7	96.2

RETRACTED

**Table 4:** Discussion of the BraTS 2018 dataset in comparison.

Techniques	Acc	Spec	Sens
Dolphin SCA+ FNB	95.3	95.3	97.7
DWT+DBN	93.20	96	95
Bayesian HSC multi-SVNN	92.56	95.09	94.29
Fine-tuned CNN	92.42	95.04	94.05
Fractional CSO	93.35	96	95
PLA + Dense Net-169	96.8	97	98

## Data Availability

The data shall be made available on request.
